RETRACTED

# Ectopic expression of ROR1 prevents cochlear hair cell loss in guinea pigs with noise‐induced hearing loss

**DOI:** 10.1111/jcmm.15545

**Published:** 2020-07-07

**Authors:** Jun Zhang, Wei Zhang, Qinliang Zhang

**Affiliations:** ^1^ Department of Children’s Rehabilitation Linyi People’s Hospital Linyi China; ^2^ Electrocardiogram Room Linyi People’s Hospital Linyi China

**Keywords:** cochlear hair cell loss, NF‐κB signalling pathway, noise‐induced hearing loss, ROR1, Wnt5a

## Abstract

Noise‐induced hearing loss (NIHL) is one of the most frequent disabilities in industrialized countries. Evidence shows that hair cell loss in the auditory end organ is responsible for the majority of various ear pathological conditions. The functional roles of the receptor tyrosine kinase ROR1 have been underscored in various tumours. In this study, we evaluated the ability of ROR1 to influence cochlear hair cell loss of guinea pigs with NIHL. The NIHL model was developed in guinea pigs, with subsequent measurement of the auditory brainstem response (ABR). Gain‐of‐function experiments were employed to explore the role of ROR1 in NIHL. The interaction between ROR1 and Wnt5a and their functions in the cochlear hair cell loss were further analysed in response to alteration of ROR1 and Wnt5a. Guinea pigs with NIHL demonstrated elevated ABR threshold and down‐regulated ROR1, Wnt5a and NF‐κB p65. The up‐regulation of ROR1 was shown to decrease the cochlear hair cell loss and the expression of pro‐apoptotic gene (Bax, p53) in guinea pig cochlea, but promoted the expression of anti‐apoptotic gene (Bcl‐2) and the fluorescence intensity of cleaved‐caspase‐3. ROR1 interacted with Wnt5a to activate the NF‐κB signalling pathway through inducing phosphorylation and translocation of p65. Furthermore, Wnt5a overexpression decreased the cochlear hair cell loss. Collectively, this study suggested the protection of overexpression of ROR1 against cochlear hair cell loss in guinea pigs with NIHL *via* the Wnt5a‐dependent NF‐κB signalling pathway.

## 1 INTRODUCTION

As a sensorineural injury, noise‐induced hearing loss (NIHL) is caused by years of accumulation of exposure to noise, primarily affecting the high‐frequency region of the auditory system, with a distinctive notch noted between 4 and 6 kHz.^1^ Hair cells within the inner ear in mammals primarily function to perceive sound and head movement while this function can be potentially damaged due to either noise exposure or by damage brought on by ototoxic drug use, which may cause permanent deficits in hearing and balance.^2^ Cochlear hair cells are generally comprised of inner hair cells as well as three rows of outer hair cells, with the inner hair cells representing the primary sensory cells, while the outer hair cells mainly function to improve the sensory performance of the cochlea, predominantly at low sound‐intensity levels.^3^ The key site of NIHL damage is in the vicinity of the outer hair cells of the cochlea, and this damage is known to be irreversible.^4^ Unfortunately, no effective therapies exist for treating the damaged cochlea. Therefore, treatment in the form of an effective therapy preventing the progression of auditory hair cell apoptosis would be greatly beneficial.^5^

RETRACTED

Receptor tyrosine‐kinase‐like orphan receptor 1 (ROR1) is an orphan‐receptor tyrosine‐kinase‐like surface antigen, rarely expressed in normal adult tissues; however, its expression has been detected in certain cases of B‐cell malignancies, cancer cells, as well as in various tissues during embryogenesis.^6^ ROR receptors are common cell surface receptors primarily involved in the processes of signal transduction, cell‐cell collaborations, as well as having a mediatory role in cell proliferation, differentiation and survival.^7^ The importance of ROR1 has been demonstrated in relation to the innervation of auditory hair cells by spiral ganglion neurons.^8^ More specifically, a missense mutation in ROR1 causes profound sensorineural hearing loss in Turkish population.^8^ ROR1 is a Wnt5a receptor that influences a range of cellular functions, including proliferation, differentiation and migration.^9^, ^10^ Wnt5a is also capable of activating the nuclear factor‐κB (NF‐κB) pathway, potentially acting to translocate the nucleus, and in doing so, activating either anti‐apoptotic or apoptotic genes.^11^, ^12^ A previous report demonstrated the protective effects of NF‐κB on noise‐induced cochlear cell loss.^13^ In addition, evidence has also been provided that the NF‐κB signalling pathway confers protection against kanamycin‐induced cochlear sensory cell loss.^14^ Therefore, based on the available literature, we hypothesized that ROR1 may affect cochlear hair cell loss, which implicated in the NF‐κB signalling pathway and Wnt5a. Furthermore, we aimed to investigate the cochlear hair cell loss through the process of promoting endogenous ROR1 in cultured cochlear hair cells obtained from the guinea pigs induced with NIHL model.

## 2 MATERIALS AND METHODS

### 2.1 Subjects

A total of 105 healthy, variegated male guinea pigs with sensitive auricles (aged 3 months, weighing 250‐350 g) were purchased from the animal experiment centre of the Union Hospital Affiliated to Tongji Medical College of Huazhong University of Science and Technology (Wuhan, Hubei, China). The guinea pig binaural eardrum integrity was confirmed by conducting an electron microscopic examination. The guinea pigs were housed in separate cages under controlled conditions with temperatures ranging between 21‐24°C, relative humidity of 40%‐60% and background noise under 50 dB sound pressure level (SPL). The 105 guinea pigs were subsequently randomly grouped as follows: normal group (normal guinea pigs, n = 15), si‐ROR1 group (normal guinea pigs treated with siRNA targeting ROR1, n = 15), si‐Wnt5a group (normal guinea pigs treated with siRNA targeting Wnt5a, n = 15), si‐NC group (normal guinea pigs treated with siRNA negative control n = 15), noise‐induced hearing loss (NIHL) group (NIHL guinea pigs without treatment, n = 15), ROR1 vector group (NIHL guinea pigs injected with ROR1 vectors, n = 15) and empty vector group (NIHL guinea pigs injected with empty vectors, n = 15).

RETRACTED

### 2.2 Animal treatment

In the normal, si‐ROR1, si‐Wnt5a and si‐NC groups, the left ear of each animal was used as the surgical ear. The siRNAs targeting ROR1 and Wnt5a as well as the NC sequences were transduced into the guinea pig cochlea through the Lipofectamine^TM^ 2000 kit (Invitrogen Inc, Carlsbad, CA, USA). The normal group was not subjected to noise exposure.

In the NIHL, ROR1 vector and empty vector groups, the left ear of each animal was selected for the operation. The ROR1 overexpression plasmid was transduced into guinea pig cochlea using the Lipofectamine™2000 kit (Invitrogen Inc). Guinea pigs in the ROR1 vector group were microinjected with 10 μL of the ROR1 vector on the left cochlea, while guinea pigs in the empty vector group were injected with an empty vector on the left cochlea.^15^, ^16^ Lipofectamine™ 2000 reagent and the ROR1 overexpression plasmid was mixed at a ratio of 3 μL: 1 μL/μg. Then, the mixture was allowed to stand at room temperature for 20 minutes followed by a microinjection to the guinea pig. The vectors used in the experiment were provided by Shanghai GenePharma Co., Ltd. (Shanghai, China). Each guinea pig was housed individually in a 20 × 20 × 20 cm cage, which was placed in a 26 m^3^ exposed chamber. The noise between 20‐2000 Hz was generated by the signal generator and amplified by a 400 W loudspeaker (GY type). A B&K 2107 frequency analyser was used to continuously monitor the exposure process, with the SPL metre (A weight) set at 110 dB, while the animals were exposed to sound within ± 1 dB of inhomogeneity of the sound field. The guinea pigs were exposed to excessive sound once a day (1.5 hours once) for seven consecutive days. The guinea pigs in the normal group were housed in a quiet environment, free of noise exposure.

### 2.3 Auditory brainstem response detection

Auditory brainstem response (ABR) was measured prior to the cochlear microinjection, prior to noise exposure (3 days after cochlear microinjection) as well as 7 days following noise exposure (before animals were euthanized) in a double‐walled, soundproof room. The guinea pigs were subsequently anaesthetized with an intraperitoneal injection with 2% pentobarbital sodium at a dose of 40 mg/kg. A one‐inch needle served as the electrode. Subdermal electrodes were inserted at the anterior fontanelle of the central cranial line, under the test ear, and at the tip of the nose (ground). An alternating polarity click was used as the primary stimulating sound. Acoustic stimuli were delivered a TDH49 earphone, which was placed approximately 1 cm away from the animal's external auditory canal. Parameters of ABR were set as the following: stimulus at 13/sec, filter band at 100‐3000 Hz, 10MS of scanning time and 1024 cycles of superimposition. The auditory response threshold was assessed by the ABR wave III reaction threshold. Body temperature was maintained in normal limits during the evaluation process.

RETRACTED

### 2.4 Immunohistochemistry

The left cochlea from guinea pigs in each group was subsequently cut into sections. Following the removal of the temporal bones, the cochlea and vestibular organs were isolated under an anatomic microscope by drilling of cochlear apex and dislocating the stapes. The cochlea was subsequently dissected, fixed, decalcified, dehydrated and ultimately cut into 4 μm paraffin embedded sections. The sections were conventionally dewaxed, hydrated and repaired using a microwave. Hydrogen peroxide was then used for the inactivation of the endogenous enzymes. After being blocked with normal goat serum, the sections were incubated with the primary antibody to ROR1 (ab135669, 1:50), Wnt5a (ab174963, 1:50), NF‐κB p65 (ab16502, 1:50) and NF‐kB p65 (phospho S276) (ab194726, 1:50) at 4°C for 24 hours. Horseradish peroxidase (HRP)‐labelled secondary goat anti‐rabbit immunoglobulin G (IgG) (ab6721, 1:1000) was subsequently added to the sections, followed by incubation at room temperature for 50 minutes. All antibodies were purchased from Abcam Inc (Cambridge, UK). In between each step, the sections were washed three times (5 min/time) with phosphate buffered saline (PBS, pH = 7.4). The sections were then coloured using diaminobenzidine (DAB, DAKO Company, Glostrup, Denmark), with the positive cells in brownish yellow, followed by a counterstaining with haematoxylin, conventional dehydration, clearing and mounting. Control incubations were routinely processed with normal goat serum as the negative control (NC). Under observation with a microscope with Corti acting as the unit, the Image‐Pm Plus image analysis system (Version 6.0.260; Olympus Optical Co., Ltd, Tokyo, Japan) was employed to detect the integrated optical density (OD) of 10 Corti fields of vision among each group. Five different high‐power fields (200×) of each section were also randomly selected for observation (100 cells per field).^17^ The percentage of positive cells (brownish yellow)/total cells > 10% was regarded as positive (+), that of positive cells < 10% was negative (−). The intensity of staining was divided into four grades (intensity scores): no staining (0 point), weak brown staining (1 point), moderate brown staining (2 points) and strong brown staining (3 points), while the percentage of positive cells was divided into four grades (percentage scores): <5% (0 point), 5%‐30% (1 point), 31%‐70% (2 points), >75% (3 points). The staining positivity was determined by the following formula: overall score = percentage score × intensity score. The overall score ≤ 3 was defined as negative, and > 3 was defined as positive.^18^

RETRACTED

### 2.5 Phalloidin‐fluorescein isothiocyanate (FITC) and propidium iodide (PI) double staining

Fixed auditory vesicles were decalcified using ethylenediaminetetraacetic acid (EDTA). The cochlea was then fixed 3‐5 times with 4% paraformaldehyde, followed by fixation in a refrigerator for up to 12 hours. The fixed cochlea was rinsed with 0.01 mol/L PBS solution followed by the complete separation of the Corti under an anatomic microscope. The Corti was rinsed 3 times with 0.01 mol/L PBS and incubated with 1% bovine serum albumin (BSA) solution containing 0.25% Triton 100 and 0.01 mol/L PBS at room temperature for 20 minutes. The Corti was rinsed 3 times and incubated with PBS containing phalloidin‐FITC (Sigma‐Aldrich Chemical Company, St Louis, MO, USA) at the ratio of 1:250 overnight at 4°C. The stained Corti was later washed with PBS and stained with 5 μg/mL PI solution (Gene‐Probe, Marlborough, MA, USA) at room temperature for 10 minutes. Afterwards, the Corti was rinsed 3 times with PBS, flattened on clean glass, sealed with 50% glycerol and ultimately observed using a confocal microscope.

### 2.6 Reverse transcription quantitative polymerase chain reaction (RT‐qPCR)

The cochlea tissues (two cochleae in each Eppendorf tube) preserved in liquid nitrogen were fully ground. In accordance with the instructions provided by the Trizol Reagent (Invitrogen Inc, Carlsbad, CA, USA), the total RNA in cochlea tissues was extracted. The reverse transcriptase system was subsequently prepared according to the reagent instructions of synthesizing cDNA. cDNA (2 μL) was taken as a template to prepare the 25 μL RT‐qPCR reaction system: 12.5 μL of 2 × Super Real Premix, 0.75 μL of 10 μmol/L forward primer, 0.75 μL of 10 μmol/L downstream primer, 9 μL of RNase‐free ddH_2_O. The PCR reaction conditions were as follows: pre‐denaturation at 95°C for 15 minutes, and 40 cycles of denaturation at 95°C for 10 seconds, annealing and extension at 60°C for 30 seconds. Following that reaction, the relative expression of mRNA was calculated by implementing a 2^−ΔCt^ method, using β‐actin as the internal reference. The experiment was repeated three times (this section of the experiment was also applicable for the cell experiments), with the RT‐qPCR primers depicted in Table 1.

RETRACTED

**TABLE 1:** The primer sequences for RT‐qPCR

Gene	Primer sequence (5’‐3’)
ROR1	Forward: CATGGGGACTTCCTGCACAT
	Reverse: AATGGGCAGCAGGGACTTAC
Wnt5a	Forward: AAGTTCGGTGCCGACTTTCA
	Reverse: AATCGTGCACCAGTCACCAA
NF‐κB	Forward: AGTTCGCGGGTACTGAGTTG
	Reverse: TATTGCCGAGCACACGAAGT
Bcl‐2	Forward: TGTGGCTGCATTCGCTCTAA
	Reverse: TGCTCTGTTTTCCTCGGTCC
Bax	Forward: GCCCTTTTGCTTCAGGGTTT
	Reverse: AGTTCGTCCCCAATTCGCTT
p53	Forward: GGTGCGTATTTCCAGGGTGA
	Reverse: TAGGGGAAGCGGGACAGTAA
β‐actin	Forward: CGAGTACATCCCCTCGCTTC
	Reverse: TTTTGCTCTGGGCTTCGTCT

Abbreviations: Bax, Bcl‐2‐associated X protein; Bcl‐2, B‐Cell CLL/Lymphoma 2; NF‐κB, nuclear factor kappa; ROR1, receptor tyrosine‐kinase‐like orphan receptor 1; RT‐qPCR, reverse transcription quantitative polymerase chain reaction.

### 2.7 Western blot analysis

Total protein was then extracted using the protein extraction kit (Bestbio Biotechnologies, Shanghai, China). The protein concentration of each sample was determined by the bicinchoninic acid (BCA) kit (23 225; Pierce, Waltham, MA, USA) and adjusted using deionized water. Next, approximately 10% sodium dodecyl sulphate‐polyacrylamide gel electrophoresis (SDS‐PAGE) gel was prepared (P0012A, Beyotime Biotechnology Co., Shanghai, China). Protein samples (50 μg) were then added to each well, treated with cycles of an electrophoresis set at a constant pressure of 80 to 120 V for 2 hours. The protein was then transferred onto the polyvinylidene fluoride (PVDF) membrane (ISEQ00010; Millipore Corp., Billerica, MA, USA) using the wet transfer method at a current of 250 mA for 90 minutes. The PVDF membrane was then blocked with Tris Buffered Saline with Tween (TBST) buffer containing 5% skim milk powder for 2 hours. After one TBST washing, the membrane was incubated with the following primary antibodies overnight at 4°C: rabbit anti‐ROR1 (#4102, 1:1000, Cell Signaling Technology, Beverly, MA, USA), Wnt5a (bs‐1948R, 1:100, Bioss Biotech, Beijing, China), NF‐κB p65 (ab16502, 1:500, Abcam Inc, Cambridge, UK), NF‐κB p65 (phospho S276) (ab194726, 1:500, Abcam Inc, Cambridge, UK), Bcl‐2 (bs‐20351R, 1:100, Bioss Biotech, Beijing, China), Bax (bs‐0127R, 1:100, Bioss Biotech, Beijing, China), p53 (bs‐8687R, 1:100, Bioss Biotech, Beijing, China), β‐actin (bs‐0061R, 1:500, Bioss Biotech, Beijing, China). The membrane was washed 3 times using TBST (10 minutes each time), incubated with the secondary antibody, horseradish peroxidase (HRP)‐conjugated goat anti‐rabbit IgG (1:2000, ab6721, Abcam Inc, Cambridge, UK) at room temperature for 1 hour, and ultimately washed 3 times with PBS/Tween 20 (PBST) (10 min/time). The membrane was coloured using the enhanced chemiluminescence (ECL) reaction solution (WBKLS0100, Millipore Corp., Billerica, MA, USA). Images were later acquired after the membrane was exposed in a dark box. With β‐actin as the internal reference, the ratio of the grey value of the target bands to those of the β‐actin bands served as the relative protein expression.

RETRACTED

### 2.8 Cell transfection and grouping

The cochlear tissues were incubated in Hank solution containing 0.25 mg/mL papain (Calbiochem‐Novabiochem, Bad Soden, Germany) at room temperature for 10 minutes, and subsequently washed two times with the Hank solution. The basilar membrane was then separated from the cochlea axis using a stainless needle under an anatomic microscope. The hair cells were added into the culture medium and adhered to the cover glass at the bottom of the petri dish. The separated hair cells were then be cultured with the Dulbecco's modified eagle's medium (DMEM) containing 100 U/mL 10% foetal bovine serum (Gibco, Carlsbad, CA, USA), penicillin and streptomycin in an incubator at 37°C with 5% CO_2_ and 95% humidity. Once the cell confluence reached 80%‐90%, cells were passaged. After 12‐24 hours, 20 μg/mL 5‐bromo‐2‐oxy‐deoxyuridine (Sigma‐Aldrich Chemical Company, St Louis, MO, USA) was added to inhibit the growth of non‐neuronal cells, with the culture medium renewed after 48 hours. The cochlea hair cells of guinea pigs in the NIHL group were transfected with different plasmids and divided into empty vector group (transfected with empty vector), siRNA‐NC group (transfected with siRNA‐NC), siRNA‐ROR1 group (transfected with siRNA‐ROR1), ROR1 vector group (transfected with ROR1 vector), siRNA‐Wnt5a group (transfected with siRNA‐Wnt5a), Wnt5a vector group (transfected with Wnt5a vector) and ROR1‐vector + siRNA‐Wnt5a group (co‐transfected with the ROR1 vector and siRNA‐Wnt5a). The full length of guinea pig ROR1 cDNA (XM_013143073) and Wnt5a cDNA (XM_013143893) were synthesized, subsequently cloned and inserted into pIRES2‐EGFP plasmids and pIRES2‐RFP plasmids. The sequences of the plasmids were confirmed with a DNA sequencing. ROR1 and Wnt5a expression vectors used for transfection were purchased from Shanghai GenePharma Co., Ltd. (Shanghai, China). Approximately 24 hours prior to their transfection, the cells were inoculated in a six‐well plate. When the cell confluence reached approximately 70%, the cochlear hair cells were transfected using a lipofectamine 2000 kit (Invitrogen Inc, Carlsbad, CA, USA). Following 6 hours of transfection, the medium was renewed, and the cells were collected for subsequent experimentation after an additional 48 hours of a culture process. The sequences designed by a web‐based online software system siDirect: ROR1 siRNA1, ROR1 siRNA2 or nonspecific control siRNA (control) purchased from Open Biosystems (Rockford, IL) were used in the experiment. The sequences of siRNA‐ROR1 were 5’‐ATGGAACATTTCAAGTGATTTTG‐3’ (siRNA1), and 5’‐TGGAACATTTCAAGTGATTTTGA‐3’ (siRNA2). The sequence of siRNA‐Wnt5a was 5’‐GTGCAATGTCTTCCAAACTCTTC‐3’.

RETRACTED

### 2.9 Immunofluorescence assay

The transfected cells were fixed with 40 g/L paraformaldehyde and reacted with 0.3% Triton X‐100 (Shanghai Solarbio Bioscience & Technology Co., Ltd., Shanghai, China) for 10 minutes, followed by a blockade using 10% BSA at room temperature for 1 hour. The cells were then incubated with the antibodies to cleaved‐caspase‐3 (diluted 1:100 with PBS, Abcam Inc, Cambridge, UK) at 4°C overnight and washed 3 times with PBS (10 minutes each time). After that, the cells were incubated with the secondary antibody, goat anti‐rabbit antibody (1:200; Abcam Inc) in dark conditions at room temperature for 1 hour. The cells were then incubated with 4',6‐diamidino‐2‐phenylindole (DAPI) solution at room temperature for 10 minutes. The immunofluorescence samples were subsequently placed in the Leica 880 fluorescence inverted microscope (LMS 800; Leica Camera AG, Solms, Germany). At least 3 fields of evenly distributed cells in each sample was collected and observed with a combination of blue and green excitation.

### 2.10 Co‐immunoprecipitation (Co‐IP) assay

The cultured cochlear hair cells were centrifuged, collected and lysed by the addition of 100‐200 μL IP lysis solution (Beyotime Institute of Biotechnology, Shanghai, China) containing protease inhibitor (Roche Company) on ice for 30 minutes. Then the cells were centrifuged at 10 000 g and 4°C for 3‐5 minutes, and the supernatant was collected. The cells were incubated overnight at 4°C with the mixture of 100 μL lysis solution and 20‐30 μL antibody by gentle shaking. Next, 30 μL Protein G (Beyotime Institute of Biotechnology, Shanghai, China) agarose beads were added into the cell lysate following overnight incubation with antibody, and incubated at 4°C for 4 hours for coupling. After IP reaction, centrifugation was carried out at 3000 rpm and 4°C for 3 minutes, with the agarose beads to the bottom of the tube and the supernatant was carefully removed, followed by washing using 1 mL of lysis buffer. Additional centrifugation was conducted and the supernatant was discarded, followed by 3‐4 times of washing. At last, 40 μL protein loading buffer was added to the precipitate, and boiled for 5 minutes. After cooling, the precipitate was analysed by Western blot analysis to verify the binding of Wnt5a and ROR1.

RETRACTED

### 2.11 Flow cytometry

Flow cytometry was conducted according to the instructions of Annexin V cell apoptosis detection kit (Beijing Biosea Biotechnology Co., Ltd., Beijing, China). Cochlear hair cells were treated with 0.01, 0.10 and 1.00 nmol/L LDM for 48 hours. The cells were centrifuged, collected and washed 2‐3 times with PBS. The cells were centrifuged at 178 × g at 4°C for 10 minutes, followed by removal of the supernatant. The cells were suspended in 150 μL Binding Buffer, then added with 10 μL Annexin V‐FITC and 5 μL PI, and allowed to react at room temperature in the dark for 15 minutes. Next, 150 μL Binding buffer was added. The fluorescence intensity was measured with a flow cytometer (Coulter Electronics Inc, Hialeah, FL, USA) and analysed using FACScan software. The results were expressed as apoptosis rate.

### 2.12 Statistical analysis

All statistical analysis was conducted in connection with the SPSS 21.0 software (IBM Corp., Armonk, NY, USA). The measurement data were presented as mean ± standard deviation. Comparisons between two groups were analysed using paired *t* test. One‐way analysis of variance (ANOVA) was used for multiple‐group comparisons, followed by a Tukey's post hoc test. *P* < 0.05 was considered to be statistically significant.

## 3 RESULTS

### 3.1 NIHL model is established successfully

Initially, to confirm that the model had been successful induced, ABR detection was performed before and after noise exposure in each group, with the data and analysis of each group displayed in Table 2. ABR detection was performed before cochlea microinjection and prior to noise exposure. The results revealed no significant differences regarding the ABR threshold of each group. After 7 days, there were no significant changes detected in the ABR threshold in the normal group (*P* > 0.05). After stimulation using white noise for a 7‐day period, in comparison with the NIHL group, the ABR threshold of guinea pigs in the ROR1 vector group decreased (*P* < 0.05); however, the ABR threshold of guinea pigs in the empty vector group showed no significant changes (*P* > 0.05). These results collectively indicated that the NIHL guinea pig model was successfully established. Moreover, hearing loss was severer in the empty vector and NIHL groups than that in the ROR1 vector group (*P* < 0.05).

RETRACTED

**TABLE 2:** ABR threshold of guinea pigs before and after noise exposure (dB SPL)

Groups	n	Before cochlear microinjection	Before noise exposure	After 7 d of noise exposure
Normal group	15	15.67 ± 1.73	16.00 ± 1.28	16.60 ± 2.97
NIHL group	15	16.03 ± 2.44	16.63 ± 2.39	63.54 ± 2.82^*&^
ROR1 vector group	15	16.15 ± 1.65	16.28 ± 2.23	46.71 ± 3.32^*#&^
Empty vector group	15	16.57 ± 2.35	16.77 ± 2.19	62.97 ± 4.27^*&^

Note

There was no noise exposure in the normal group. The data were expressed as mean ± standard deviation. The data before and after noise exposure were compared by paired *t* test. One‐way analysis of variance was used for data comparison between multiple groups ^*^, *P* < 0.05 vs. the normal group; ^#^ *P* < 0.05 vs. the NIHL group; ^&^ *P* < 0.05 vs. before noise exposure.

Abbreviations: ABR, auditory brainstem response; NIH, noise‐induced hearing loss; ROR1, receptor tyrosine‐kinase‐like orphan receptor 1.

In addition, we divided normal guinea pigs into normal, si‐ROR1, si‐Wnt5a and si‐NC groups. ABR detection was performed before and after cochlear microinjection (Table S1). The results showed no significant difference in ABR threshold between the guinea pigs in each group. After microinjection, compared with the normal group, the ABR threshold of the si‐NC group had no significant change (*P* > 0.05), but the ABR threshold of the si‐ROR1 and si‐Wnt5a groups showed an increase (*P* < 0.05). Furthermore, after microinjection, the ABR threshold of the si‐ROR1 and si‐Wnt5a groups increased significantly versus pretreatment results (*P* < 0.05). Thus, ROR1 and Wnt5a may be involved in the pathogenesis of hearing loss, and ROR1 might prevent NIHL progression.

### 3.2 Down‐regulated ROR1, Wnt5a and NF‐κB in outer hair cells of cochlear tissues is associated with NIHL

Next, we employed immunohistochemistry to determine the positive expression of ROR1, Wnt5a and NF‐κB p65 in the outer hair cells of cochlear tissues of the NIHL models. Figure 1 illustrates the positive expression of ROR1, Wnt5a and NF‐κB p65 in the cochlea of the normal group without noise exposure and the cochlea of the NIHL, ROR1 vector and empty vector groups after 7 days of noise exposure. The ROR1, Wnt5a and NF‐κB p65 positive cells all had dark brown staining located in the cytoplasm and cell membrane. After seven days of noise exposure, the positive rates of ROR1, Wnt5a and NF‐κB p65 in cochlea tissues of the NIHL, ROR1 vector and empty vector groups were significantly lower than those detected in the normal cochlear tissues without noise exposure (*P* < 0.05). The ROR1 vector group presented significantly higher positive rate of ROR1, Wnt5a and NF‐κB p65 in cochlear tissues than that in the empty vector group (*P* < 0.05). The results suggested that ROR1, Wnt5a and NF‐κB p65 protein expression had been down‐regulated in the outer hair cells of cochlear tissues of the NIHL guinea pig model.

RETRACTED

**FIGURE 1:** ROR1, Wnt5a and NF‐κB p65 positive expression is at a low level in the outer hair cells of cochlear tissues of the NIHL guinea pig models. Guinea pigs with NIHL were treated with ROR1 vector or empty vector. (A) the immunohistochemical staining of ROR1, Wnt5a and NF‐κB p65 in the outer hair cells of cochlear tissues (scale bar = 25 μm); (B) the statistical analysis of panel A. The data are presented as a mean ± standard deviation. One‐way ANOVA is performed for multiple‐group comparison. ^*^ *P* < 0.05 vs. the normal group; ^#^ *P* < 0.05 vs. the empty vector group. n = 15

### 3.3 Overexpression of ROR1 inhibits the expression of pro‐apoptotic factors in guinea pigs with NIHL

RT‐qPCR and Western blot analysis were performed to measure the expression of ROR1, Bax, p53, Bcl‐2, Wnt5a and NF‐κB with the purpose of further analysing the effects of ROR1 on cochlear hair cell apoptosis. The results (Figure 2) demonstrated that, in comparison with the normal group, the NIHL group had significantly increased mRNA and protein expression of Bax and p53 (*P* < 0.05); however, there was significant decrease in the mRNA and protein expression of ROR1, Wnt5a, NF‐κB and Bcl‐2 (all *P* < 0.05). In comparison with the empty vector group, the ROR1 vector group exhibited notably diminished mRNA and protein expression of Bax and p53 (*P* < 0.05), and significantly increased mRNA and protein expression of ROR1, Wnt5a, NF‐κB and Bcl‐2 (all *P* < 0.05). The aforementioned results suggested that overexpressed ROR1 could promote the expression of Wnt5a, NF‐κB and Bcl‐2, while simultaneously inhibiting the expression of Bax and p53.

**FIGURE 2:** Up‐regulation of ROR1 decreased the expression of pro‐apoptosis genes (Bax, p53) in guinea pig cochlea but elevated the expression of anti‐apoptosis gene (Bcl‐2). Guinea pigs with NIHL were treated with ROR1 vector or empty vector. (A) the mRNA expression of ROR1, Bax, p53, Bcl‐2, Wnt5a and NF‐κB in cochlear tissues determined by RT‐qPCR. (B and C) the protein expression of ROR1, Bax, p53, Bcl‐2, Wnt5a and NF‐κB in cochlear tissues measured by Western blot analysis. The data are presented as a mean ± standard deviation. One‐way ANOVA is performed for multiple‐group comparison. ^*^ *P* < 0.05 vs. the normal group; ^#^ *P* < 0.05 vs. the empty vector group. n = 15

RETRACTED

### 3.4 Overexpression of ROR1 inhibits cochlear hair cell apoptosis in vitro

To further study the effects of ROR1 on cochlear hair cells, we first knocked down the expression of ROR1 in cultured cochlear hair cells. RT‐qPCR and Western blot assay showed that, compared with the siRNA‐NC group, siRNA‐ROR1#1 and siRNA‐ROR1#2 can significantly reduce the expression of ROR1 (Figure 3A‐B). In addition, the knockdown efficiency of siRNA‐ROR1#2 was more obvious, which was used in subsequent experiments.

**FIGURE 3:** Up‐regulation of ROR1 inhibits cochlear hair cell apoptosis in vitro. Cochlear hair cells were transduced with ROR1 vector or siRNA‐ROR1. (A) the ROR1 mRNA levels in cochlear hair cells in response to transfection of siRNA‐ROR1#1 and siRNA‐ROR1#2 assessed by RT‐qPCR. (B) the ROR1 protein levels in cochlea hair cells in response to transfection of siRNA‐ROR1#1 and siRNA‐ROR1#2 assessed by Western blot analysis. (C) the mRNA expression of ROR1, Bax, p53, Bcl‐2 in cochlear hair cells assessed by RT‐qPCR. (D and E), the protein bands and expression of ROR1, Bax, p53, Bcl‐2 in cochlear hair cells evaluated by Western blot analysis. (F) apoptosis of cochlear hair cells in the scatter plots, where the upper left quadrant indicates the necrotic cells (annexin V−/PI+), the upper right quadrant shows late apoptotic cells (annexin V+/PI+), the lower left quadrant shows live cells (annexin V−/PI−), and the lower right quadrant shows the early apoptotic cells (annexin V+/PI−). G, the percentage of early and late apoptotic cells. H, immunofluorescence staining of cleaved‐caspase‐3 (scale bar = 50 μm). The experiment was independently repeated three times. The data are presented as a mean ± standard deviation. One‐way ANOVA is performed for multiple‐group comparison. ^*^ *P* < 0.05 vs. the empty vector group; ^#^ *P* < 0.05 vs. the siRNA‐NC group

RT‐qPCR and Western blot analysis methods were applied to detect the expression of apoptosis‐related genes in cochlear hair cells (Figure 3C‐E). Compared with the empty vector group, the ROR1 vector group displayed significantly decreased mRNA and protein expression of Bax and p53, however, marked increases in mRNA and protein expression of ROR1 and Bcl‐2 were detected (*P* < 0.05). Compared with the siRNA‐NC group, the siRNA‐ROR1 group had significantly elevated mRNA and protein expression of Bax and p53, but significantly decreased mRNA and protein expression of ROR1 and Bcl‐2 (*P* < 0.05).

The effect of ROR1 on the cell apoptosis of cochlear hair cells was evaluated based on the flow cytometry analyses of Annexin V‐FITC/PI double staining (Figure 3F‐G). The results showed that compared with the empty vector group, the ROR1 vector group had a significantly reduced apoptosis rate (*P* < 0.05), while the apoptosis rate of the siRNA‐ROR1 group was significantly higher than that of the siRNA‐NC group (*P* < 0.05).

RETRACTED

Besides, the expression of cleaved‐caspase‐3 was detected using immunofluorescence assay (Figure 3H). The results showed that cleaved‐caspase‐3 was localized in the cytoplasm of the mesenteric cells. The fluorescence intensity of cleaved‐caspase‐3 in the ROR1 vector group was significantly higher than that in the empty vector group, while the fluorescence intensity of cleaved‐caspase‐3 in the siRNA‐ROR1 group was significantly lower than that in the siRNA‐NC group (*P* < 0.05). Taken together, these results indicated that the up‐regulation of ROR1 could inhibit the cell apoptosis of cochlear hair cells.

### 3.5 ROR1 activates NF‐κB p65 signalling pathway by interacting with Wnt5a in cochlear hair cells

Having confirmed that overexpression of ROR1 in cochlear hair cells could up‐regulate the expression of Wnt5a and activate the NF‐κB signalling pathway, we next tested for any interaction between ROR1 and Wnt5a. First, the immunofluorescence assay in Figure 4A showed that ROR1 and Wnt5a co‐localized in the cytoplasm of cochlear hair cells, suggesting that there might be an interaction between them. As shown in Figure 4B, the Co‐IP assay validated the interaction between ROR1 and Wnt5a. The results of Western blot analysis (Figure 4C) showed that overexpression of ROR1 or Wnt5a induced p65 phosphorylation. Notably, overexpression of Wnt5a did not affect the expression of ROR1. Furthermore, the phosphorylation level of p65 was decreased following both overexpression of ROR1 and Wnt5a knockdown. Overexpression of ROR1 or Wnt5a decreased the protein expression of Bax while elevating Bcl‐2 protein expression. However, co‐treatment with ROR1 overexpression and Wnt5a knockdown increased Bax protein expression yet decreased Bcl‐2 protein expression. These results indicated that ROR1 inhibited apoptosis of cochlear hair cells via Wnt5a‐dependnet NF‐κB signalling pathway activation.

**FIGURE 4:** ROR1 mediates NF‐κB p65 expression by interacting with Wnt5a in cultured cochlear hair cells. (A) co‐localization of ROR1 and Wnt5a assessed by immunofluorescence assay (scale bar = 25 μm). (B) the interaction between ROR1 and Wnt5a assessed by Co‐IP assay. (C) the protein expression of ROR1, p‐p65, p65, Bax and Bcl‐2 in response to the treatment of ROR1 vector, siRNA‐ROR1 or Wnt5a vector + ROR1 vector evaluated by Western blot analysis. The experiment was independently repeated three times

RETRACTED

### 3.6 Overexpression of ROR1 inhibits cochlear hair cell apoptosis through the activation of the NF‐κB signalling pathway by binding to Wnt5a in vitro

Next, we sought to explain the effects of Wnt5a on cochlear hair cells. We first knocked down the expression of Wnt5a in cochlear hair cells. RT‐qPCR and Western blot assay showed that, compared with the siRNA‐NC group, siRNA‐Wnt5a#1 and siRNA‐Wnt5a#2 can significantly reduce the expression of Wnt5a (Figure 5A‐B). In addition, the knockdown efficiency of siRNA‐Wnt5a#2 was more obvious, which was used in subsequent experiments.

**FIGURE 5:** Overexpression of ROR1 inhibits cochlear hair cell apoptosis through the activation of the NF‐κB signalling pathway by binding to Wnt5a in vitro. Cochlear hair cells were transduced with ROR1 vector, siRNA‐ROR1 or Wnt5a vector + ROR1 vector. (A) the Wnt5a mRNA levels in cochlear hair cells in response to transfection of siRNA‐Wnt5a#1 and siRNA‐Wnt5a#2 assessed by RT‐qPCR. (B) the Wnt5a protein levels in cochlea hair cells in response to transfection of siRNA‐Wnt5a#1 and siRNA‐Wnt5a#2 assessed by Western blot analysis. (C) the mRNA protein of related genes in cochlear hair cells tested by RT‐qPCR. (D and E) the protein bands and expression of related genes in cochlear hair cells evaluated by Western blot analysis. (F) apoptosis of cochlear hair cells in the scatter plots in which the upper left quadrant shows the necrotic cells (annexin V−/PI+), the upper right quadrant shows the late apoptotic cells (annexin V+/PI+), the lower left quadrant shows the live cells (annexin V−/PI−), and the lower right quadrant shows the early apoptotic cells (annexin V+/PI−). (G) the percentage of early and late apoptotic cells. (H) immunofluorescence staining of cleaved‐caspase‐3 (scale bar = 50 μm). The experiment was independently repeated three times. The data are presented as a mean ± standard deviation. One‐way ANOVA is performed for multiple‐group comparison. ^*^ *P* < 0.05 vs. the empty vector group; ^#^ *P* < 0.05 vs. the siRNA‐NC group; ^&^ *P* < 0.05 vs. the siRNA‐ROR1 + empty vector group

RT‐qPCR and Western blot analysis were used to detect the expression of apoptosis‐related genes in cochlear hair cells (Figure 5C‐E). Relative to the empty vector group, the Wnt5a vector group had significantly lower mRNA and protein expression of Bax and p53 (*P* < 0.05); however, significantly increased mRNA and protein expression of Wnt5a, Bcl‐2 and NF‐κB were observed (*P* < 0.05). Compared with the siRNA‐NC group, the siRNA‐Wnt5a group had significantly increased mRNA and protein expression of Bax and p53 (*P* < 0.05), but significantly decreased mRNA and protein expression of Wnt5a, Bcl‐2 and NF‐κB (*P* < 0.05). Compared with siRNA‐ROR1 + empty vector group, the siRNA‐ROR1 + Wnt5a vector group exhibited a significantly lower mRNA and protein expression of Bax and p53 (*P* < 0.05), while significantly higher mRNA and protein expression of Wnt5a, Bcl‐2 and NF‐κB (*P* < 0.05) were observed.

RETRACTED

The effect of ROR1 and Wnt5a on cochlear hair cell apoptosis was assessed using flow cytometry analysis of Annexin V‐FITC/PI double staining. The results (Figure 5F‐G) showed that compared with the empty vector group, the Wnt5a vector group had a significantly decreased apoptosis rate (*P* < 0.05), with the apoptosis rate of the siRNA‐Wnt5a group was significantly higher than that of the siRNA‐NC group (*P* < 0.05). Compared with the siRNA‐ROR1 + empty vector group, the siRNA‐ROR1 + Wnt5a vector group displayed a significantly lower apoptosis rate (*P* < 0.05).

Furthermore, the expression of cleaved‐caspase‐3 was detected using immunofluorescence assay (Figure 5H). The results showed that cleaved‐caspase‐3 was localized in the cytoplasm of the mesenteric cells. The fluorescence intensity of cleaved‐caspase‐3 expression in the Wnt5a vector group was significantly higher than that in the empty vector group, and that in the siRNA‐Wnt5a group was significantly lower than that in the siRNA‐NC group. Compared with the siRNA‐ROR1 + empty vector group, the siRNA‐ROR1 + Wnt5a vector group had significantly higher fluorescence intensity of cleaved‐caspase‐3 expression.

All in all, the data suggested that overexpression of ROR1 could up‐regulate Wnt5a, and that up‐regulation of Wnt5a led to activation of the NF‐κB signalling pathway, which acts to inhibit the apoptosis of cochlear hair cells.

## 4 DISCUSSION

NIHL represents a perpetual hearing impairment commonly resulting from a continued exposure to high levels of noise.^3^ Currently, there are no effective therapies for preventing or restoring hearing loss caused by noise exposure (NIHL).^19^ The present study investigated the effects of ROR1 on the regulation of hair cell apoptosis in the cochlea of guinea pigs, providing evidence that ROR1 inhibited cochlea hair cell apoptosis by activating the NF‐κB signalling pathway via Wnt5a, thereby mitigating NIHL.

Observations obtained in this study demonstrated that ROR1 and Wnt5a expression decreased in the NIHL cells. ROR1 is known to belong to the receptor tyrosine kinases (RTKs) primarily involved in various cellular processes such as differentiation, proliferation, migration, angiogenesis, survival and cell interactions.^20^, ^21^ ROR1 knockdown has been reported to lead to malfunctioned hair cell innervation as well as atypical cochlear development.^8^ Wnt5a, a typical ligand that activates the β‐catenin‐independent pathways, is implicated in numerous diseases including cancers, metabolic disorders and inflammatory diseases.^22^ A previous study showed that the Wnt5a expression was significantly decreased in Cmah‐null mouse in association with the age‐related hearing loss.^23^ The data of the current study indicated that ROR1 could up‐regulate the expression of Wnt5a and promote the activation of the NF‐κB signalling pathway. ROR1 commonly functions as a Wnt5a receptor, proactively regulating the activation of NF‐κB in leukaemia B cells as well as in the cochleae.^24^ Wnt5a is a crucial ROR1 ligand, most notably involved in the ROR1‐dependent signalling pathway, and acting as a promoter to cancer cell growth.^25^ A previous study demonstrated that the basal Wnt5a‐Fz5 signalling pathway was a supporter of macrophage survival, aiding in the maintenance of innate immune functions via the transcriptional activation of NF‐κB (p65), which in turn proves to be a central factor by which p65 can sustain Wnt5a expression.^26^ A previous study conducted by Nagy *et al* argued that the NF‐κB signalling pathway was overexpressed in the cochlea, and also suggested that p65 was expressed in the nuclei of the hair cells, acting to support the cells in the p5 rat organ of Corti.^27^

RETRACTED

We also demonstrated in this study that the overexpression of ROR1 could up‐regulate Wnt5a, which in turn led to activation of the NF‐κB signalling pathway, thus acting to inhibit the apoptosis of cochlear hair cells. Wnt5a has also been found to bind to ROR1, and these two proteins were commonly co‐transfected in 293 cells to promote activation of the pleiotropic transcription factor NF‐κB.^28^ In addition, we also observed that ROR1 and Wnt5a together inhibited cell apoptosis by an indirect effect on anti‐apoptotic genes, including that of Bcl‐2 and pro‐apoptotic genes, such as Bax, p53, and cleaved‐caspase‐3. Currently, a consensus exists suggesting that most of the important factors relayed in the mediation of cell apoptosis can be targeted by specific therapeutic strategies. Chief among these are Bcl‐2 proteins, the gatekeepers of the mitochondrial pathway, caspases, the executioner enzymes or the so‐called endogenous caspase inhibitors.^29^ In addition, caspases, particularly caspase‐3, have drawn attention due to their involvement in the nerve growth factor‐induced programmed cell death in the development of the inner ear.^30^ Furthermore, a previous study stressed the proposal that overexpression of Wnt5a could down‐regulate caspase‐3^31^ while another prior study showed that silencing Wnt5a increased Bcl‐2 expression and decreased Bax expression, consistent with the findings in this study.^32^ Finally, Wier *et al* demonstrated that the NF‐κB anti‐apoptotic gene transcription could modulate cell apoptosis through a caspase‐3 produced p65 fragment.^33^

RETRACTED

## 5 CONCLUSIONS

In conclusion, the key data presented by this study provide evidence suggesting that ROR1 represses cochlear hair cell apoptosis in guinea pigs with NIHL by activating Wnt5a. These findings indicate that ROR1 can be used as a therapeutic target of NIHL prevention, thus offering new insights possibly informing novel therapeutic approaches for treating NIHL. Certainly, it would be of interest to investigate further the molecular mechanism underlying the ROR1 regulation of Wnt5a, with an aim to develop a clinical trial.

## CONFLICT OF INTEREST

The authors declare that they have no competing interests.

## AUTHOR CONTRIBUTION

**Jun Zhang:** Conceptualization (equal); Methodology (equal); Visualization (equal); Writing‐review & editing (equal). **Wei Zhang:** Data curation (equal); Investigation (equal); Software (equal); Validation (equal). **Qinliang Zhang:** Formal analysis (equal); Resources (equal); Supervision (equal); Writing‐original draft (equal).

## ETHICAL STATEMENTS

The study was conducted in strict accordance with the *Guide for the Care and Use of Laboratory Animals* of the National Institutes of Health. The applied protocols were approved by the Institutional Animal Care and Use Committee of Linyi People's Hospital.

## Supporting information

Table S1

## Data Availability

Research data not shared.
